RETRACTED

# Doppler Ultrasound Imaging Combined with Fetal Heart Detection in Predicting Fetal Distress in Pregnancy-Induced Hypertension under the Guidance of Artificial Intelligence Algorithm

**DOI:** 10.1155/2021/4405189

**Published:** 2021-10-08

**Authors:** Su Liu, Yue Sun, Na Luo

**Affiliations:** ^1^Department of Obstetrics, The Third Affiliated Hospital of Qiqihar Medical College, Qiqihar 161000, Heilongjiang, China; ^2^Department of Ultrasound, The Third Affiliated Hospital of Qiqihar Medical College, Qiqihar 161000, Heilongjiang, China

## Abstract

This study was to improve the feasibility and economic benefits of intelligent medical system Doppler ultrasound (DUS) imaging technology combined with fetal heart detection to predict the fetal distress in pregnancy-induced hypertension (PIH), so as to reduce the risk of deterioration of the patient's condition. The characteristics of DUS images were analyzed, and a diffusion filter reducing the specificity was adopted to improve the smooth speckle noise of DUS images. 120 pregnant women in hospital were the subjects of the study, all of whom received ultrasound cord blood flow testing and fetal heart monitoring. 88 PIH patients with fetal distress were diagnosed and included in the observation group, and 32 healthy pregnant women tested during the same period were identified as the control group. Clinical data were reviewed and analyzed. The diagnostic rates of fetal distress by simple fetal heart monitoring and DUS detection combined with fetal heart monitoring were compared. The results showed that 26.7% of fetal distress were diagnosed by fetal heart monitoring alone, and 73.3% of fetal distress were diagnosed by combined testing, so the diagnostic accuracy of the combined detection method was greatly higher than the single fetal heart detection (*P* < 0.05). The Pulsatility index (PI), resistance index (RI), and *S*/*D* values detected by the umbilical artery in the observation group were 1.48, 0.85, and 4.31, respectively. The PI, RI, and *S*/*D* values detected by the umbilical artery in the control group were 0.96, 0.64, and 3.59, respectively. The results of arterial detection were significantly higher than those of the control group, and the difference was of significant scientific significance (*P* < 0.05). In summary, the PI and RI values of the middle cerebral artery (MCA) detected by DUS diagnosis can effectively reflect the current status of the fetus in the uterus and reduce the mortality of the fetus. The images guided by DUS imaging technology can clearly show the current status of the fetus in the uterus, effectively improve the medical diagnostic efficiency, and have important reference value for the development of intelligent medical equipment.

RETRACTED

## 1. Introduction

Fetal distress is a relatively common complication in the perinatal period of pregnant women, and it is a syndrome of fetal life safety due to hypoxia and acidosis in the womb. The incidence rate is about 5.0%, and the incidence is high in late pregnancy, especially in high-pregnancy pregnant women, which can lead to low fetal intelligence, damage to the nervous system, cerebral palsy, and even perinatal death in severe cases [1]. In the past, clinical detection of fetal distress mainly used fetal heart detection, but there are many interference factors, and false positive results often appear in clinical practice, which seriously affects the judgment and evaluation of doctors, so the accuracy of fetal distress detection appears very important [2]. In recent years, many studies have found that color Doppler ultrasound (DUS) has a significant diagnostic effect, and color Doppler ultrasound combined with fetal heart detection of fetal distress has a high clinical value.

DUS technology has many advantages such as nonionizing radiation and noninvasiveness, so it has been widely used in various fields of medicine in the 1940s. The original DUS technology is two-dimensional DUS, which can only reflect the situation in the tissue in a planar state. With the development of DUS imaging technology, color DUS was born, and portable high-resolution DUS probes are widely used clinically [3, 4]. Some scholars apply the matching tracking algorithm to ultrasonic Doppler noise processing, and the ultrasonic signal changes rapidly. The algorithm proposed by Mallat can well reflect local information and reduce noise relatively objectively and fairly. Some scholars also introduced an algorithm based on adaptive decomposition to perform time-frequency analysis on the signal, using the traditional discrete wavelet transform algorithm and wavelet packet transform algorithm to denoise the DUS blood flow signal, and the clarity of the image was well improved. Fetal heart rate detection is also more accurate. Fetal heart detection plays an important role in the diagnosis of the fetus, and it can reflect the fetal heart function of the fetus, which is regulated by the central nervous system [5, 6]. Whether or not the fetus is in good condition can be monitored by electronic fetal heart rate, which can effectively diagnose whether the fetus is hypoxic [7].

DUS image is a kind of real-time image with better imaging effect on blood vessels and soft tissues. Under the guidance of DUS, there is no need to operate, and the patient can be accurately observed locally through images. With the continuous development of computer technology and image recognition technology, artificial intelligence (AI) is widely used in the medical field [8]. AI is a branch of computer science, including intelligent technology, simulation, and extension. It can imitate human thoughts and behaviors, and learn and solve problems. AI has brought about great convenience in finance, games, medicine, health, etc. AI can rapidly, safely, and effectively integrate the information, which has brought disease diagnosis and treatment into a new era [9, 10]. DUS image guidance has a higher success rate than touch-based guidance, and it has been proven in the medical field. Traditional fetal heart detection has also begun to develop in the direction of Internet monitoring and intelligent diagnosis [11]. Fetal detection can clearly reflect the functional status of the fetus. In terms of low price and use, fetal heart detection is the preferred method of fetal detection [12]. DUS imaging can observe the shape of the fetus, but it cannot show whether the fetus is hypoxic or distressed. The fetal heart detection combined with DUS can clearly observe the shape of the fetus and it can also understand whether the fetus is hypoxic, so that predicting fetal distress is more accurate. Traditional ultrasound images are widely used in the detection of certain biological characteristics, mainly for the detection of fetal growth parameters, such as the measurement of amniotic fluid, head circumference, abdominal circumference, biparietal diameter, and placental maturity, but this method is too complicated, and its detection and diagnosis are time-consuming. The image definition is relatively low, and the resolution is not high. The color Doppler ultrasound scanner has high fidelity quality for pregnant women's uterine artery, renal artery, fetal brain, etc., in the hemodynamic detection of fetal blood circulation.

RETRACTED

Therefore, the pregnant women with fetal distress were selected as the research objects, and the meaning of pregnancy-induced hypertension (PIH) with fetal distress was predicted based on AI algorithm DUS imaging and fetal heart detection. In addition, the selected AI medical automatic system was tested to obtain certain DUS image characteristics. The algorithm can effectively present the fetal distress situation, and provide a reference basis for clinically ensuring the diagnosis rate of fetal distress and the clinical diagnosis of fetal distress.

## 2. Methods

### 2.1. Research Objects

Hundred and twenty pregnant women hospitalized in our hospital from 2018 to 2020 were taken as the study subjects. All of them received ultrasound cord blood flow testing and fetal heart monitoring. 88 PIH patients with fetal distress were diagnosed and included in the observation group, and 32 healthy pregnant women tested during the same period were identified as the control group. The age range of the research subjects was 23–36 years old (an average age of 28.6 ± 0.5 years old). All pregnant women were first babies and their menstrual conditions were normal before conception. There was no obvious difference in clinical data of all pregnant women (*P* > 0.05), and they can be compared.

The inclusion criteria were defined as follows: patients who were pregnant, with 37–41 weeks of gestational age, no age limit, single fetus, and no obvious abnormalities in the obstetric examination; all patients who conformed to the diagnostic index of fetal distress; and patients with clinical manifestations of headache, edema, and higher blood pressure concentration. The subjects voluntarily participated in this study.

The exclusion criteria were defined as follows: women with gestational age less than 37 weeks; women with bad multiple births; women without routine obstetrics; and women with pregnancy complications. Of all the 120 patients enrolled in the group, 88 cases of fetal distress were detected as the observation group, and 32 healthy pregnant women who were examined at the same time were the control group. The difference in clinical data of patients was not statistically great (*P* > 0.05). This trial had been endorsed by the ethics committee of the hospital, and all patients and their families had given informed consents and signed the informed consent forms.

### 2.2. Detection Methods

All pregnant women were examined with a color DUS diagnostic apparatus. Pregnant women were required to be in supine position, and the probe frequency was 2–6 MHz. The abdomen of pregnant women was scanned using a probe to find the umbilical artery, and the images were analyzed with the appropriate obstetric analysis software. In the process of maternal umbilical artery measurement, any umbilical cord can be selected to test the blood flow frequency. The double top diameter measurement section of tire head can be selected for translation probe downward. The measurement of middle cerebral artery (MCA) can very well show the fetal basilar artery ring, which was positioned in the middle of the cerebral artery, and the blood flow spectrum can be obtained. The cross section of the cranium can be obtained. The side of the cerebral cortex was selected to detect the flow frequency of the cerebral artery. The blood flow probe can display the beginning of the renal artery beside the left and right veins of the spine in the transverse section of the abdomen, and the Doppler blood flow spectrum can be obtained based on the sampling of the renal artery. The sampling volume of the color DUS measurement was 2 mm, which corrected the angle between the sampling volume and the blood vessel. The Doppler was adjusted to the same direction as the blood flow to obtain at least 3 complete and clear pulse Doppler blood flow images. After the above operations were repeated more than 5 times for each indicator, there was a relatively stable frequency map, and then the measurement was carried out. The DUS instrument had its own calculation program, and the calculation results and images were all analyzed offline. S represented the maximum end-systolic arterial blood flow velocity of the pregnant woman, *D* represented the end-diastolic blood flow velocity of the pregnant woman, and *S*/*D* was the ratio of the peak value of the end-systolic arterial blood flow to the end-diastolic blood flow velocity. Pulsatility index (PI) = (*S* − *D*)/average blood flow velocity value and resistance index (RI) = (*S* − *D*)/*S*.

RETRACTED

The diagnostic criteria for DUS were abnormal changes in fetal heart rate. Amniotic fluid above 80 mm indicated too little amniotic fluid; if the heart rate was higher than 160 beats per minute or lower than 120 beats per minute, it was determined as tachycardia or bradycardia; if the umbilical artery of the fetus was above 3.00 or MCA was below 1.08, it showed abnormal DUS frequency; and if the fetal movement decreased or disappeared gradually, it showed abnormal fetal movement.

### 2.3. Research on the Core Issues of Imaging Computer-Assisted Interventional Surgery Navigation

Advanced surgical medical image processing technology combined with computer AI to participate in medical operations can not only better complete disease diagnosis but also clearly show the shape and characteristics of the fetus in the uterus.  Figure 1 shows that the research issues affecting navigation mainly included image processing technology and computer-assisted technology. At this stage, the three-dimensional visualization of medical images, the three-dimensional segmentation of medical images, and preoperative and postoperative operations were all key issues in medical operations.

### 2.4. Collection and Preprocessing of DUS Images

As shown in Figure 2, DUS images processing included image acquisition, image preprocessing, horizontal view processing, longitudinal view processing, and precise positioning of puncture. The system firstly started with image acquisition (including horizontal scanning and vertical scanning), and performed denoising and binarization preprocessing on the DUS video stream collected by the patient to obtain the DUS image of the pregnant woman. In the horizontal false case measurement system, the DUS view was processed in the longitudinal direction. The rough positioning was performed, then the DUS probe was converted, and the horizontal view was processed. The image position would also change as the probe position moved up and down. In the scanned Google image, the horizontal scanning image was separated to accurately locate the position of the fetus in the womb. The GUI module can directly display the processing process, thereby realizing real-time guidance to the physician.

RETRACTED

The DUS instrument adopted the DW series B-type DUS diagnostic instrument (DW-3101B, Xuzhou Dawei Electronic Equipment Co., Ltd.), as shown in Figure 3(a). Figure 3(b) is an electronic convex array probe. The DUS instrument can not only perform real-time dynamic aperture imaging, dynamic emission point-by-point focusing, dynamic digital filtering but also digital control frequency scanning, digital enhancement, and point correlation and other image processing technologies. In addition to saving a large number of images, it can replay and view many images after diagnosis, and it also has a variety of functions of body marking and subtitle annotations.

DUS images collection included vertical scanning and horizontal scanning. When scanning, the scanning depth of the DUS probe was 8–10 cm, and then the sacrum was moved along the midline. The DUS video stream was collected at 15 frames per second, with 10–20 s each time. The DUS probe was placed in the gap between L3 and -L4, the probe was switched to scan at the same video stream speed, and the patient was scanned vertically and horizontally. After the scan was completed, the image was stored in the computer via universal serial bus (USB), and DUS images processing can be performed offline.  Figure 4(a) is an image of horizontal scan, and Figure 4(b) is an image of vertical scan.

### 2.5. Block Diagram of the System

Figure 5 shows the flowchart of DUS longitudinal view processing system. Starting with automatic recognition, it can use the support vector machine (SVM) supervised learning mode to perform the automatic recognition. If the detection target was recognized, the panoramic mode of the nano image started to record the spinous process structure, and the most suitable image stitching module was performed through quality evaluation. After the level of the spinous process was identified, it was divided in the panoramic image, and the DUS system was then projected into the original DUS image. The lateral view processing system had to separate the interspinous process image from the image.

### 2.6. DUS Horizontal View Recognition Process

The DUS horizontally processed image was preprocessed to obtain a binarized DUS image, and the image was classified and then normalized to perform feature extraction on the image. The feature extraction here was mainly for images between spinous processes, and the traditional extraction algorithm was mainly for matching values, vertebral bodies, black pixels, and external cavity positions. As shown in Figure 6, the image was preprocessed, and then feature extraction was performed. The images were classified using a classifier to separate the interspinous process image, and then the target that needed to be identified was identified accurately.

RETRACTED

### 2.7. Processing of DUS Images

Random speckle noise was a limitation of DUS images, caused by the interference of the scattering of uneven fine tissues. Due to the presence of noise, the spatial resolution and the interpretability of the image were reduced. Speckle noise was not conducive to the recognition of the image by the naked eye, and it concealed the effective features extracted by the image, so it was particularly important to effectively denoise the image. In this study, a better image denoising model was adopted, so the speckle noise was multiplicative noise and related to the image signal:

(1) $$\begin{array}{c} f\left(a,\;b\right)=\;g\left(a,\;b\right)\cdot \delta m\left(a,\;b\right), \end{array}$$

where *f*(*a*, *b*) represented the original image with noise, *g*(*a*, *b*) represented the uncertain noise-free image, and *δm*(*a*, *b*) referred to the multiplicative noise.

Image speckle noise was also called multiplicative noise.

Robust nonlinear diffusion is the physical process of balancing the concentration. The diffusion equation is a fluctuation of material density diffusion. The image was denoised using a nonlinear partial differential equation, and the equation was shown as follows:

(2) $$\begin{array}{c} \frac{\xi H\left(x,y,t\right)}{\xi H}=\mathrm{div}\left[C\left(\left\|\nabla H\right\|\right)\cdot \nabla H\right],\\ H\left(t=0\right)=H0, \end{array}$$

where ∇ represented the gradient operator, div was the divergence operator, ||∇*H*|| referred to the gradient of the image *H*, *C*(*x*) was the diffusion coefficient, and *H*0 represented the original image.

There was a certain functional relationship between the gradient magnitude and the diffusion coefficient. ||∇*H*|| approached positive infinity, then *C*(*x*) approached 0; and the large magnitude value spread and tended to be gentle, it may be the edge; and if the small gradient value tended to the smoothing, there may be areas of image noise.

Effective nonlinear diffusion is very important for the attenuation of speckle noise, and the Tukey dual-weight error norm can increase the robustness of the algorithm. The equation was as follows:

(3) $$\begin{array}{c} \alpha \left(x,\psi \right)=\left\{\begin{array}{c} x\cdot \left[1-{\left(\frac{x}{\psi }\right)}^{2}\right],\;\left|x\right|\leq \psi ,\\ 0, \end{array}\right. \end{array}$$

where Ψ was the scale factor, and the robust error norm was introduced to analyze the performance of the *α* function. After the optimization criterion, the robust nonlinear diffusion formula was given as follows:

(4) $$\begin{array}{c} \frac{\partial \mu }{\partial t}=\mathrm{div}\left[\alpha \left(\left|\nabla \mu \right|\right)\cdot \left(\left|\nabla G\left(\delta \right)*\mu \right|\right)\cdot \frac{\nabla \mu }{\left|\nabla \mu \right|}\right], \end{array}$$

where *|*∇*G*(*δ*)*∗μ|* represented the gradient value of the Gaussian low-pass filtered image with the standard deviation *δ*, which substituted the gradient value ∇*μ* of the original image, and the robustness of sensitive noise was effectively enhanced.

RETRACTED

There are many algorithms for image denoising quality, and each algorithm has different DUS images denoising. The quality standards are evaluated according to objective evaluation criteria. The equation was as follows:

(5) $$\begin{array}{c} \mathrm{MSE}=\frac{1}{\mathrm{MN}}\sum_{m=0}^{M-1}\sum_{n=0}^{N-1}{\left[I\left(m,n\right)-\hat{I}\left(m,n\right)\right]}^{2}, \end{array}$$

(6) $$\begin{array}{c} \mathrm{SNR}=10\log_{10}\frac{1/\mathrm{MN}\sum_{m=0}^{M-1}\sum_{\text{n}=0}^{N-1}I^{2}\left(m,n\right)}{\mathrm{MSE}}, \end{array}$$

(7) $$\begin{array}{c} \mathrm{PSNR}=10\log_{10}\frac{255^{2}}{\mathrm{MSE}}. \end{array}$$

In equations (5), (6), and (7), MSE was the mean square error, SNR referred to the input signal-to-noise ratio, PSNR represented the peak signal-to-noise ratio, and the edge retained the parameter *f* measurement. In addition, I referred to the original image, $\hat{I}$ was the image denoised by the algorithm, MN referred to the image size, and 255 was the order of magnitude.

The *f* measurement criteria were defined as follows:

(8) $$\begin{array}{c} \phi =\frac{\sum_{m=0}^{M-1}\sum_{n=0}^{N-1}\left[\Delta I\left(m,n\right)-\bar{\Delta }I\right]\left[\Delta \hat{I}\left(m,n\right)-\bar{\Delta }\hat{I}\right]}{\sqrt{\sum_{n=0}^{N-1}{\left[\Delta I\left(m,n\right)-\bar{\Delta }I\right]}^{2}{\left[\Delta \hat{I}\left(m,n\right)-\bar{\Delta }\hat{I}\right]}^{2}}}. \end{array}$$

In equation (8), Δ meant that the image was subjected to a high-pass filter, which was realized by a 3 × 3 Laplacian operator; $\bar{\Delta }$ was the average value of the Laplacian operator and the image after convolution. The smaller the MSE, the more similar the evaluated image was to the original image, and it also showed that the algorithm was applied well. The larger the *φ* value, the better the performance of the algorithm in evaluating the preservation of image edges.

RETRACTED

The image contrast was enhanced through morphological transformation. Firstly, two disc structure elements with a radius of 3 were established. After the top hat and the bottom hat, Rt and Rb, respectively, were obtained, and R0 and Rc were obtained by opening and closing operations, the equation for the brightening part of the top hat image was expressed as follows:

(9) $$\begin{array}{c} \mathrm{Rb=Rt-Rc}. \end{array}$$

After the bottom hat was transformed, the image after the opening operation was subtracted to get the dark part of the image:

(10) $$\begin{array}{c} \text{Rd}=\text{Rb}-\text{R0.} \end{array}$$

Finally, the bright area of DUS images was enhanced, and the dark area was weakened. The calculation equation was as follows:

(11) $$\begin{array}{c} \text{Rn}=\text{Rf}\alpha -\text{Rd}+\alpha \text{Rb.} \end{array}$$

The adaptive binarization algorithm improved the interpretability of the image, and the image obtained by calculation can realize the segmentation of the object and the image background. The higher the threshold of the image area, the higher the image brightness, and the smaller the threshold of the image area, the lower the image brightness.

The threshold was calculated using the following equation:

(12) $$\begin{array}{c} q\left(a,b\right)=\left\{\begin{array}{c} 1,g\left(a,b\right)<P\left(a,b\right),\\ 0, \end{array}\right. \end{array}$$

where *q*(*a*, *b*) was a binarized image and the threshold *T*(*a*, *b*) was calculated by the following equation:

(13) $$\begin{array}{c} P\left(a,b\right)=m\left(a,b\right)\left[1+v\frac{\gamma \left(a,b\right)}{1-\gamma \left(a,b\right)}-1\right]. \end{array}$$

In the above equation, *m*(*a*, *b*) was the local average and *γ*(*a*, *b*) represented the local average deviation.

(14) $$\begin{array}{c} \gamma \left(a,b\right)=g\left(a,b\right)-m\left(a,b\right). \end{array}$$

*V* was a deviation that can control the change of the threshold, and the adaptation level of the threshold can be adjusted according to the *V* value.

If the size of the image area was the same, then *g*(*a*, *b*) = *m*(*a*, *b*); if *p*(*a*, *b*) and *m*(*a*, *b*) were both 0, *g*(*a*, *b*) became the background color.

### 2.8. Statistics and Analysis

The SPSS22.0 software was adopted for the statistical processing of experimental data. Continuous variables were expressed as mean ± standard deviation ($\bar{x}\pm S\;D$), and an independent sample *t*-test was used for difference comparison. Binary variables were represented by percentage (%) data, and chi-square test was used for difference comparison. When *P* < 0.05, the difference between groups was considered to be statistically significant.

RETRACTED

## 3. Results

### 3.1. Image Analysis

In this study, the robust nonlinear diffusion was adopted. All images were collected in the same environment and operated by the same physician. The image processing software platform was MATLABR2015a, the hardware platform computer memory was 4G running (2.53 GHz Core(TM)i3 CPU), and the cropped image size was 330 × 290.  Figure 7(a) is the original image, and Figure 7(b) is a robust nonlinear diffusion image.

### 3.2. Diagnosis Rate of Fetal Distress

As illustrated in Figure 8, 32 cases (26.7%) of fetal distress were diagnosed by fetal heart detection (mode A) alone, and 88 cases (73.3%) were diagnosed by combined detection (mode B). The combined detection method was greatly higher than that of fetal heart detection alone (*P* < 0.05).

### 3.3. Test Results of RI, PI, and S/*D*

Figures 9–11 show the results of PI, RI, and *S*/*D*. The RI of the umbilical artery in the control group was 0.64 and the cerebral artery was 0.83. The RI test result of the umbilical artery in the observation group was 0.85, and that in the cerebral artery was 0.46. The PI of the umbilical artery in the control group was 0.96 and that in the cerebral artery was 1.92. The PI test result of the umbilical artery in the observation group was 1.48, and that in the cerebral artery was 0.91. The *S*/*D* of the umbilical artery of the control group was 3.59, and that in the cerebral artery was 3.99. The *S*/*D* test result of the umbilical artery in the observation group was 4.31, and that of the cerebral artery was 2.51. The results of PI, RI, and *S*/*D* detected by the umbilical artery of the observation group were significantly higher than those of the control group, and the difference was significant (*P* < 0.05).

## 4. Discussion

Fetal distress is a high-risk pregnancy disorder in obstetrics and gynecology. Acute hypoxia can easily cause neonatal cerebral palsy and hypoxic ischemic encephalopathy [13, 14]. Fetal heart detection is a physical detection method to detect whether the fetal body is functioning well. It can make a good prediction of the health of the fetus in the womb of a pregnant woman, and it can also effectively observe the fetal movement in the case of uterine contractions [15, 16]. The application of AI medical system in DUS images processing reduces the incidence of clinically unsafe accidents. In this study, AI algorithms were applied to DUS images of medical systems to analyze the characteristics of DUS images. After classification and sorting, the image feature extraction characteristics were normalized. The algorithm ignores the difference in image intensity and independently recognizes the interpretability of DUS images. In addition, a diffusion filter reducing the specificity was applied to improve the smooth speckle noise of DUS images. Many domestic literatures report that fetal heart detection and cord blood flow measurement can predict fetal distress well [17]. Morales-Roselló et al. [18] used DUS to study the brain-placental ratio, and the results showed 10% of fetal fetal heart abnormalities, with some being suitable for detection by cardiopulmonary resuscitation. Some scholars have also used contrast-enhanced ultrasound to distinguish benign and malignant thyroid nodules. The ultrasound images of primary malignant lymphoma of the thyroid (PTL) showed a uniform increase in the overall size, a larger lesion volume, and blood flow signals in the nodules. Based on visible signals, the study of Cantisani et al. [19] proved that elastography was of great value in the identification of benign and malignant thyroid glands. In this study, the diagnosis rate of fetal heart detection alone was 26.7%, and the diagnosis rate of combined intelligent DUS detection was 73.3%, so the combined detection method showed much higher diagnosis accuracy in contrast to the fetal heart detection alone (*P* < 0.05). In the results of PI, RI, and *S*/*D* in this study, the RI of the umbilical artery in the control group was 0.64, and that of the cerebral artery was 0.83. The RI test result of the umbilical artery in the observation group was 0.85, and that of the cerebral artery was 0.46. The PI of the umbilical artery in the control group was 0.96 and that of the cerebral artery was 1.92. The PI test result of the umbilical artery in the observation group was 1.48, and that of the cerebral artery was 0.91. The *S*/*D* of the umbilical artery of the control group was 3.59, and that of the cerebral artery was 3.99. The *S*/*D* test result of the umbilical artery in the observation group was 4.31, and that of the cerebral artery was 2.51. The value of S/D test result of the umbilical artery in the observation group was significantly higher than the control group.

RETRACTED

The fetal distress caused by PIH is clinically believed to be the main cause of fetal hypoxia in the uterus. Under normal circumstances, after the uterine placenta is implanted, the surrounding blood circulation will change with the extension of the pregnancy time. When the placenta matures, the capillaries will increase and the resistance around the blood vessels will decrease, thereby promoting blood flow; and as the amount rises, it can provide more oxygen to the fetus [20]. When PIH appears, the whole body of the pregnant woman will experience spasm of small arteries, the permeability of the blood vessels will increase, causing the vascular exudation to increase, and the blood will be concentrated; then, the pregnant woman will be in a hypercoagulable state. As PIH continues to worsen, the volume of red blood cells and blood viscosity increases, and the degree of vascular occlusion also increases, which will cause hypoxia, and the fetus will not be able to breathe normally. Color DUS can help doctors better evaluate the condition of the fetus, check the increase in the *S*/*D* value of the umbilical artery in time, and combine the conditions of MCA and renal artery to reflect whether the resistance in the placenta is too high, which can reflect whether the fetus is ischemic and hypoxic [20]. Research results show that the diagnosis rate of prenatal DUS fetal distress in uterus is 97.6%, indicating that the early detection of fetal hypoxia in uterus enables timely effective measures to reduce the fetal mortality rate. The results of PI, RI, and *S*/*D* detected by the umbilical artery in the observation group of this study were observably higher than those in the control group, indicating that DUS combined with fetal heart detection can effectively predict PIH fetal distress.

## 5. Conclusion

In order to improve the efficiency of fetal distress detection for pregnancy-induced hypertension, this research applied intelligent algorithms to Doppler ultrasound images to detect patients with pregnancy-induced hypertension. Then, a robust nonlinear diffusion filter was selected to preprocess the image to improve the efficiency of PIH fetal distress detection. It turned out that DUS scanning can automatically detect and filter image features under the application of an intelligent system. The images guided by the DUS imaging technology can clearly show the current status of the fetus in the uterus, which effectively improved the medical diagnostic efficiency. The MCA PI, RI, and other values of the color DUS diagnosis can effectively reflect the current status of the fetus in the uterus and reduce fetal mortality. However, the algorithm analysis selected in this study cannot completely eliminate the image speckle noise. In the follow-up work, how to completely eliminate speckle needs in-depth study, expand the sample size, and ensure the wide application of the system. Doppler ultrasound images based on artificial intelligence algorithms can show pregnancy-induced hypertension, effectively improve the efficiency of medical diagnosis, and have important reference value for the development of intelligent medical equipment.

RETRACTED

In short, the results of this study can provide a theoretical basis for improving the prediction of PIH fetal distress in the DUS image combined with fetal heart detection in the intelligent medical system.[21].

## Figures and Tables

**Figure 1:** Schematic diagram of the core problems of imaging computer-assisted interventional surgery navigation.

**Figure 2:** The block diagram for DUS images processing.

**Figure 3:** Diagram of DUS diagnostic equipment. (a) Ultrasound Diagnostic System. (b) Convex array probe.

**Figure 4:** DUS scan images.

**Figure 5:** The flowchart of DUS longitudinal view processing system.

**Figure 6:** DUS recognition process of intrauterine fetal lateral view.

**Figure 7:** Ultrasound image comparison.

**Figure 8:** Comparison on diagnosis rate of fetal distress. *Note*. A refers to result using the fetal heart detection alone; B shows the result of combined detection method. ^*∗*^ indicates that the difference was statistically obvious (*P* < 0.05).

**Figure 9:** PI test results of umbilical arteries and cerebral arteries in the two groups. ^*∗*^ indicates that the difference was statistically obvious (*P* < 0.05).

**Figure 10:** RI test results of umbilical arteries and cerebral arteries in the two groups. ^*∗*^ indicates the difference was statistically obvious (*P* < 0.05).

**Figure 11:** *S*/*D* test results of umbilical arteries and cerebral arteries in the two groups. ^*∗*^ indicates that the difference was statistically obvious (*P* < 0.05).

## Data Availability

The data used to support the findings of this study are available from the corresponding author upon request.
